# Neurotransmitters and Electrophysiological Changes Might Work as Biomarkers for Diagnosing Affective Disorders

This article has been retracted.

**DOI:** 10.1155/2021/9116502

**Published:** 2021-09-18

**Authors:** Fei Liang, Rou Feng, Simeng Gu, Shan Jiang, Xia Zhang, Naling Li, Minghong Xu, Yiyuan Tang, Fushun Wang

**Affiliations:** ^1^Institute of Brain and Psychological Science, Sichuan Normal University, Chengdu, Sichuan 610000, China; ^2^Department of Psychology, Jiangsu University, Zhenjiang, Jiangsu 212013, China; ^3^Department of Neurology, Lianyungang Hospital of Chinese Medicine, Nanjing University of Chinese Medicine, Lianyungang, China; ^4^Department of Psychological Sciences, Texas Tech University, Lubbock, TX 79409, USA

## Abstract

Affective disorders are the leading causes of human disability worldwide; however, the diagnosis is still hard to define, because emotion is the least study subjects in psychology. Recent emotional studies suggest that human emotions are developed from basic emotions, which are evolved for fundamental human lives. *Even though most psychologists agree upon the idea that there are some basic emotions, there is little agreement on how many emotions are basic, which emotions are basic, and why they are basic*. In our previous papers, we suggested that there are three basic emotions: joy, fear, and disgust. *These basic emotions depend on the peptides and monoamines: dopamine-joy (peptides-reward), norepinephrine-fear (anger), and serotonin-disgust (sadness)*. Further tests with event-related potentials (ERP) found that joy, fear, and disgust showed the fastest response compared with other emotions, suggesting that they are fast automatic responses, which confirmed that these three emotions are prototypical emotions. Other basic emotions, anger and sadness, are due to object induced behaviors instead of sensation of object, so they developed secondary to prototypical emotions. Thus, we concluded that only joy, fear, and disgust are prototypical emotions, which can mix into other emotions, like the primary colors. In all, the neural substrates for all emotions, including the affections, are possibly monoamine neuromodulators: joy-dopamine (peptides), fear (anger)–norepinephrine, and disgust-serotonin. We hope these basic emotional studies will offer some neural mechanisms for emotional processing and shed lights on the diagnosis of affective disorders.

## 1. Introduction

Affective disorders are the leading causes of disability worldwide; for example, major depressive disorders are affecting more than 17% of the general population [1]. The neural mechanisms of the affective disorders (such as depression, anxiety, and functional neurological disorders) are yet to be uncovered [2, 3]. The best way to study the affective disorders is through the basic emotional theory, which suggested that basic emotions are due to monoamines and peptides [4, 5]. A widespread assumption in emotional theories is that human emotions are developed from a limited number of basic emotions, which are called *basic*, *primary*, or *fundamental emotions* [6–8]. These basic emotions are developed at the phylogenetically and ontogenetically primary stage and were evolved to handle fundamental life tasks [9], such as finding something to eat (joy), avoiding being eaten (fear), or avoiding toxic food (disgust). Basic emotions are developed early in evolution to cope effectively with changing environmental demands [10]. They can activate the body to deal with prototypical situations that have significant implications for survival, and they are fairly common to all animal species as they interact with their external environment, with conspecifics, and with members of other species [11]. In addition, these basic emotions cannot be broken down further into more basic psychological components [12]. Basic emotion theory is a plausible approach that has stimulated a number of empirical lines of research (e.g., in the context of facial expression detection, neuroimaging studies, and evolutionary psychology) [13]. Nevertheless, basic emotion theory has recently been criticized by some researchers, because many studies about basic emotions have met some troubles in differentiating the basic emotions (such as *fear*, *anger*, *joy*, *sad*, and *disgust*) with distinct universal signals, especially the localization of the central nervous system [14]. For example, neuroimaging data were found to be inconsistent with specific one-to-one correspondence between fMRI localization and behavioral measurements of basic emotions. It is suggested by Barrett that “to date, no consistent and specific one-to-one correspondence has been observed between physical measurements and anger, sadness, fear, disgust etc” [13]. These data have led to controversy about basic emotions and posed significant challenges to the theory of basic emotions.

The reason for the complications might be due to the fact that “basic emotions” used in these measurements are not “basic” enough, and these emotions can be further divided into even more primary emotions [15]. Even though most psychologists agree upon the idea that there are some basic emotions, there is little agreement about how many emotions are basic, which emotions are basic, and why they are basic. For example, Waston (1930) (refer to [6]) proposed three basic emotions: *fear*, *love*, and *rage*; Panksepp (1982) (refer to [6]) proposed four: *expectancy*, *fear*, *rage*, and *panic*; Shaver (1987) (refer to [6]) proposed five: *fear*, *sadness*, *anger*, *joy*, and *love*; and Johnson-Laird and Otaley (1989) (refer to [6]) also proposed five: *happiness*, *sadness*, *fear*, *anger*, and *disgust* [6]. Yet others proposed an even greater number; Ekman proposed six basic emotions: *fear*, *anger*, *joy*, *sadness*, *surprise*, and *disgust*; Plutchik (1980), Tomkins (1984), and Izard (1977) (refer to [15]) respectively suggested that there are eight, nine, and ten basic emotions [15]. Recently, a study by Jack et al. on facial expressions found that anger and disgust appear very similar in that they share a wrinkled nose, and fear and surprise are similar in that they share raised eyebrows, so they proposed four basic emotions: *joy*, *sadness*, *fear*, and *anger* [16]. Previously, we proposed three basic emotions: *joy*, *sadness*, and *fear* (*anger*). We took fear and anger as one emotion or two sides of the same coin, because fear and anger are both due to the “fight-or-flight” response, which is a function of the locus ceruleus norepinephrine system [15].

Although these theories may differ, they all posit the existence of basic emotions. However, there is no consensus about the number of real basic emotions, let alone the reasoning for categorization as basic emotions. Arnold (1960) proposed that emotions are object-directed [17]. Lazarus suggested that “emotion is not psychologically meaningful unless it is related to an object” [18]; emotion is perceived as part of an object itself rather than one's reaction to it [19]. Emotion is similar to the color, which is a feature of an object, but it is perceived by the eye. In order to explore the basic emotions empirically, many researchers have extrapolated basic emotions with facial expressions. Basic emotions are developed phylogeneticaly and ontogenetically at the stage when facial expression has not been developed, so it is necessary to screen the basic emotions with objects instead of facial expressions. So in this paper, we used object pictures to screen six widely accepted basic emotions.

## 2. Results

### 2.1. Only Three Basic Emotions Can Be Elicited by Object Pictures

Thirty one college students (19 females, 12 males, all right handed, aged 18-22 years, mean 19.6 ± 1.4) provided written informed consent and participated in the study. Object pictures from the International Affective Picture System (IAPS) and the Chinese Affective Picture System (CAPS) were used. The criteria for choosing pictures were that only objects were shown on the picture and neither complicated scenery, human facial pictures, nor words were included. In order to avoid ambiguity of responses, pictures with only one featured object, such as a snake, cake, or fly, were preferred. 170 pictures (100 from IAPS and 70 from CAPS) were pooled together. Joy accounted for 29.4 ± 2.7% of responses, fear for 15.3 ± 1.4%, disgust for 12.0 ± 1.7%, sadness for 1.3 ± 1.2%, surprise for 2.5 ± 1.1%, and anger for 1.5 ± 1.8%, and neutral responses accounted for 38.0 ± 3.1% (Figure 1(a)). The vast majority of object-evoked emotional responses in this study were *joy*, *fear*, and *disgust*. Sadness, surprise, and anger were seldomly selected as responses.

Then, we calculated the accuracy rate for each picture. Pictures were categorized according to the emotion that gained more than half of the responses, and we found that 48 pictures can be categorized as joy, 31 as disgust, 34 as fear, and 57 as neutral emotions, but none of the pictures elicited a greater than 50% response rate of anger, surprise, or sadness (Figure 1(b)). The accuracy rates for these categorized pictures were 67.3 ± 5.1% for neutral, 76.5 ± 3.9% for joy, 55.4 ± 3.7% for fear, and 71.4 ± 4.3% for disgust (Figure 1(c)). The highest error rate for pictures categorized as anger was 4/31. The highest error rate for those categorized as sadness was 5/31, and the highest error rate of the surprise group was 6/31. The average error rates were 5.9 ± 3.7% for sadness, 3.5 ± 4.8% for anger, 4.3 ± 4.1% for surprise (*n* = 5). The distributions of chosen emotions among the pictures are shown in Figure 1(d). From the error rates of the six emotions among the pictures, we found that fear is often mixed with anger or surprise, disgust is often mixed with sadness, and neutral responses are often mixed with joy.

### 2.2. The Three Prototypical Emotions Showed the Fastest Reaction Time

Ekman declared that basic emotions should occur quickly, before one is even aware that they have started, and he said that quick onset is fundamental for the adaptive value of basic emotions [8]. Lazarus also suggested that the basic emotions were processed by the subcortical brain areas, and reaction should be automatic and faster [18]. So we compared the reaction times (RTs) for these pictures. The process was performed using a “Winner-takes-all” approach, wherein one class is classified against all others. The procedure is shown in Figure 2(a).

We added 20 pictures for sadness, anger, and surprise, respectively, in addition to object pictures. During the process of adding pictures, we found it difficult to elicit sad/angry responses from object pictures without human involvement. This may be due to the fact that sadness arises from failure or loss with no hope of reinstating the goal [19, 20], and anger arises from failure with the possibility of goal reinstatement (i.e., the goal is still possible with additional effort) [21]. *Indeed, sadness and anger are related to human behaviors instead of objects themselves*. It was difficult to select “surprise” pictures as well, so we intentionally distorted images such as elongating some animals' necks.

We first tested the error rates for the six groups of pictures, and the results showed that they exhibited reasonable accuracy (Figure 2(b)), 76.5 ± 3.9% for joy, 55.4 ± 3.7% for fear, 71.4 ± 4.3% for disgust, 69.4 ± 4.3% for surprise, 66.2 ± 4.9% for sadness, and 51.5 ± 4.6% for anger. Next, we tested the RTs, and as expected, the RTs for joy, fear, and disgust were significantly faster than those of sadness and surprise (*p* < 0.01, *F*(1, 30) = 51.3, *ŋ*^2^_*p*_ = 1.12). The averaged times were 1235.3 ± 31.4 ms for joy, 1313.7 ± 49.4 ms for disgust, 1475.3 ± 45.9 ms for fear, 2215.8 ± 61.3 ms for sadness, 2500.3 ± 53.1 ms for anger, 2837.7 ± 83.1 ms for surprise, and 1455.5 ± 77.3 ms for neutral (*n* = 31 persons) (Figure 2(c)).

We next used the 20 best categorized pictures for each emotion (the pictures that got the highest accuracy) and used the “go/no-go protocol” to test the RTs (Figures 2(d) and 2(e)). The participants only had two choices, e.g., fear or neutral. 20 new participants were recruited (11 females, 9 males). The experiments showed that RTs were 731.5 ± 28.5 ms for joy, 717.7 ± 32.8 ms for fear, 609.3 ± 29.4 ms for disgust, 1109.8 ± 31.8 ms for anger, 1489.3 ± 29.1 ms for sadness, 1283.7 ± 23.6 ms for surprise, and 985.5 ± 31.3 ms for neutral (*n* = 20). These data again demonstrated that RTs for joy, disgust, and fear are significantly faster than those of sadness, anger, and surprise (*p* < 0.01, one-way ANOVA).

### 2.3. The Three Prototypical Emotions Show the Fastest Reaction in ERP

It is important to understand the temporal dynamics of emotion processing [20]. Lazarus said “I distinguished two modes of appraisal: one automatic, unreflective, and unconscious; the other deliberate and conscious” [18]. Izard suggested that one important feature of basic emotion is automaticity: “when the event matches one of the prototype situations, the associated emotion is elicited automatically” [22]. We then adopted the event-related potential (ERP) technique, which offers excellent temporal resolution in the range of milliseconds. The protocol was the same as before (shown in Figure 2(e)), and 20 best pictures for each emotion were used and mixed randomly, and 20 participants were asked to decide if the target emotion was categorized.

Previous reports showed that fear facial expression induced significant higher response in N17, which is an early negative-going potential over occipito-temporal regions. Consistently, ERP data demonstrated that emotional objects were analyzed rapidly and affected cortical processing at very short latencies [23]. In this study, we found that objects can show even earlier response on P1 at occipito-temporal regions (Figure 3(a)). The averaged amplitudes for each emotion at P1, P2, and P3 were analyzed, which showed the amplitudes for the six emotions were significantly different (*F*(1, 20) = 58.4, *p* < 0.001, *ŋ*^2^_*p*_ = 0.92) for P1, with joy, fear, and disgust being the highest. There were no significant differences among the groups for P2 (*F*(1, 20) = 3.5, *p* = 0.025). For P3, the amplitudes were significantly different among the groups (*F*(1, 20) = 8.7, *p* < 0.01 for P3) (Figure 3(b)). Further Bonferroni-corrected pairwise comparisons for each component showed that amplitude of anger and neutral was different at P3 (*t* = 5.95, *p* < 0.01), while the difference between the amplitude of disgust with neutral was not significant (*t* = 1.95, *p* = 0.08, Figure 3(b), right). Consistent with previous reports [21], fear, joy, and disgust showed the highest effects at P1 on ERP response (Figure 3(c)). We compared the RTs for the highest relative peaks [relative peak = (categorized − neutral)/neutral], and found that the RTs were 119.3 ± 9.8 ms for joy, 123.8 ± 11.5 ms for fear, 136.9 ± 16.2 ms for disgust, 315.8 ± 21.3 ms for anger, 341.4 ± 18.7 ms for surprise, and 454.9 ± 22.4 ms for surprise (*n* = 20 subjects, Figure 3(c)). This is consistent with what Ekman suggested that the basic emotions started in a matter of milliseconds after a stimulus [8].

The response topology at P1 is shown in Figure 4(a), which also showed that joy, fear, and disgust induced the earliest responses at the occipital regions (Pz). This means the prototypical emotions are processed quickly. Dimensional emotional theory proposes that emotional states differ fundamentally along a small number of factors, e.g., valence and arousal. The IAPS were a collection of pictures with standard on valence and arousal. This is advantageous because there is no bias towards different discrete emotions. So after the EEG recordings, all participants underwent a self-report session to check the arousal and valence for all the pictures, including the 20 pictures added for anger, surprise, and sadness. No time constraint or RT was recorded; rather, accuracy was emphasized so as to warrant response reliability and maximal attention from the subjects to their own feelings. Twenty participants were asked to mark the emotions on the dimensions with valence and arousal (-4–4 for valence, 0-9 for arousal). Typical recordings from 10 people are shown in Figure 4(b). We quantified difference in emotional experience along categorical and dimensional models by computing the self-report ratings for the emotional states (Figure 4(c)). The results showed that sadness and disgust are clustered together at the negative valence, and fear and anger are often clustered together at the highest arousal. Similar to our hypothesis reported before [24], fear, anger, joy, and sadness are the basic emotions, and they represent typical example of basic emotions according to different theories, and they occupy the endpoints on the dimensional spectrum of emotions, with fear and anger along the arousal dimension and with joy opposed to sadness on the valence dimension.

## 3. Discussion

### 3.1. There Are Three Most Prototypical Emotions

This study suggests that there may be three prototypical basic emotions (joy, fear, and disgust), which is consistent with our hypothesis about the “three primary color model” of basic emotions [24, 25]. In our previous model, we suggested that there are three primary basic emotions, and these prototypical emotions are joy, fear, and disgust, which are subsided by monoamines and peptides: dopamine-joy (peptide-reward), norepinephrine-fear (anger), and serotonin-disgust (sadness). The serotonergic innervation of the brain originates primarily in the dorsal raphe nucleus of the brain stem, likely norepinephrine neurons in the locus coeruleus. These monoamines are modulated by many peptides, such as substance P, oxytocin, adrenocorticotropic hormone, vasopressin, endorphin, neuropeptide Y [4, 26]. These peptides might be the second message after monoaminergic neuromodulators or the downward pathway for monoaminergic neuromodulators.

It is proposed five criteria for basic emotions, including evolutionary significance, ontogenetic/phylogenetic primacy, cross-culture (species) universality, differentiated autonomic patterns, and the integration of social relations, emotions, and physiological processes. From this criteria, we can make the following conclusions.

*First, these prototypical emotions are evolutionarily significant.* Joy, fear, and disgust are evolutionarily the most primitive emotions and were selected because they serve primary survival functions. They serve two primary needs of human or animals: physiological need (valence) and safety needs (arousal). If the object fulfills physiological need, people like it (joy), and if not, people dislike it (disgust); if the object is expected (e.g., a traffic light at a familiar and busy intersection), a neutral response is elicited, and if the object is not expected (e.g., a tiger in the street), people will feel scared. Animals in the wild have two major tasks to survive: seeking food to eat (avoiding toxic food) and avoiding being eaten. Therefore, joy, disgust, and fear should be the most prototypical emotions. Similarly, Darwinian proposition, which can also be found in Plutchik's psycho-evolutionary theory of emotion, suggested that joy is for the need to survive and reproduce, while fear is for the need for protection [27]. In addition to joy and fear, animals might have developed another function: avoiding toxic food (disgust); for example, mushrooms have posed greater threat to the human species than spiders and snakes combined, but people do not feel fear towards mushrooms but rather disgust [28].

*Second, these prototypical emotions are automatic*. Ortony (1990) proposed that the emotions indicate something about the world [6]. The perception can happen in unconscious, automatic ways, and also in conscious ways (Figure 5). Most appraisal theorists only consider the extended appraisal (the conscious cognition or subjective emotions), but basic emotions majorly focused on the automatic appraisal (or perception) [29]. Ekman et al. said Lazarus is the only appraisal theorist who incorporates basic emotions in his framework and describes the prototypic events for basic emotions [10]. The prototypical emotions derived from the very primary sensation at an object. Barrett (2013) named this process the “conceptual act,” which is a kind of unconscious process that they automatically and effortlessly using previous knowledge to predict current sensations [13].

*Third, prototypical emotions are very fast*. Ekman et al. suggested that basic emotions were defined as a relatively brief and intense state in reaction to a specific experience [10], or basic emotions occur with a rapid onset, through automatic appraisal, with an involuntary physiologic response. The reactions are too fast to be consciously perceived. This may be the reason for James-Lange theory of emotion that “we are sad because we cried; we are scared because we run” [25]. Fear, in particular, can impact survivability only if it occurs promptly. Consistent with our data, a recent study by Costa and colleagues supports the ideas that fear, joy, and disgust were processed earlier than other emotions [21].

*Fourth, prototypical emotions are due to sensation about object*. Ekman said all emotions differ in the stimulation events, appraisals, behavioral response, and physiological responses [8]. Or emotions can be induced by reactions at different stages from Sensation–Opinion (automatic perception)–Reactions (automatic physiological changes and behavioral reactions) (S-O-R) (Figure 5). James and Lange suggested that the perception of these bodily changes is what is called an emotion [25]. Of note, a sense or perception in and of itself is not an emotion; only if the sensation results in an inherent appraisal that triggers physiological changes and behavioral reactions is an emotion [28]. People can use the physiological symptoms to feel emotions, such as dizziness at high height for fear, or nausea toward vomitus for disgust, or arousal at a sexual nude body for joy. However, people will not use the sense of an object to feel anger, although people might be angry about somebody's misbehavior; in addition, people will not feel sad if a sports game is still happening, but they may experience sad when it is over. Thus, anger and sadness are not prototypical emotions.

*Fifth, prototypical emotions are the origins of all other emotions*. The prototypical emotions are primary emotions, and they are the basis of all other emotions. The three prototypical emotions might work like the three primary colors to form all other kinds of emotions [24]. At the sensation (S) level of “S-O-R,” people can have three kinds of perceptions about an object: like (joy), dislike (disgust), or danger (fear), which represent three poles of the emotional dimensions (Figure 4(c)). At the opinion (“O”) level of “S-O-R,” people can make the appraisal of the way an object appears, such as unexpected (a bear in the zoo) or controllable (e.g., a snake in a bottle). Arnold (1960) proposed that emotions are object directed, and there are three kinds of appraisal of an object: the desirability of the object, the availability of the object, and the difficulty in getting the object [30]. These appraisals will induce “surprise” that affects the tensity of the prototypical emotions (a bear in the zoo will not induce fear, while a bear on the street will induce fear). At the behavior (“R”) level of “S-O-R,” people feel aroused at the ways of behavioral reactions (if it is expected or not, e.g., a driver drives unexpected). Every object has two features: whether it fits our needs (like or dislike) and whether it appears as expected (safety) [15].

*Sixth, prototypical emotions can be shared with animals*. Plutchick (1980) suggested that humans and all other mammals have the same basic emotions [25]. Levenson proposed two emotional systems; one is largely hard-wired and nonmodifiable in response to experience; the other is exquisitely sensitive to learning. The first one is fairly common to all animal species as they interact with their external environment, with conspecifics, and with members of other species [8]. Prototypical emotions are evolved to detect a small number of prototypical situations that have profound implications for the organism's immediate well-being and long-term survival, and they share a number of features in common with emotional systems in infrahuman species [8]. Panksepp suggested that animals might have emotions, but their emotions might be different from those of humans [29]. The animals may not experience emotions consciously, but they do experience the prototypical emotions and exhibit stereotypical behavioral reactions. Behaviorists tried to study behaviors using emotion-induced physiological changes such as saliva in Palov's dog and other behavior changes by Skinner's pigeon at a reward or punishment. *The behaviorists used three kinds of unconditional stimuli: reward (food)*, *punishment (electricity)*, *and toxic fluid (quinine)* [25], *which might be similar to the three prototypical emotions (joy*, *fear*, *and disgust)*. Therefore, our hypothesis suggests that *animal emotions (at least lower level animals*, *such as invertebrate animals) consist of just the prototypical emotions, while human emotions can also include subjective feelings* (Figure 5).

*Seventh, prototypical emotions might share the same neural basis in all the animal filed*. Many studies are searching the neural basis for basic emotions [31, 32], and it is suggested that all animals and humans should share the same specific structure for specific basic emotion. However, the brains of the insects are much different from the brains of the vertebrates. Darwin said even the insects can show certain kinds of emotions with special kinds of flight [25]. We suggested that the insects and the vertebrate share same neurotransmitters, such as dopamine, serotonin, and norepinephrine [25]. Dopamine and peptides are known to contribute to the reward system (joy) [33, 34], norepinephrine is known to contribute to the fight-or-flight response (fear) [35], and serotonin in the intestine is known to be involved in disgust [36, 37]. So dopamine, norepinephrine, and serotonin might be the basis for all emotions, and they can be combined in various degrees to produce other emotions, much like the three primary colors [24]. And their levels in blood might be used to diagnose certain affective disorders, such as anxiety and depression.

### 3.2. Other Emotions Are Derived from Prototypical Emotions

*Anger might be derived from fear*. Nearly everybody who postulates basic emotions includes *anger*, *happiness*, *sadness*, and *fear* in his list [38]. And anger appears on almost all lists of basic emotions because anger appears to be exhibited by many species, which has led many researchers to conclude that anger is a biologically basic emotion. Anger arises from failure with the possibility of goal reinstatement (i.e., the goal is still possible with additional effort), or anger occurs when the person blames some objects or agents for that thwarting [18]. An important component of anger is the desire or the tendency to fight against the agent who is blamed for what has happened. Anger is a natural response to perceived threats, and it is suggested that anger cannot be separated from those responsible for flight, so flight and fight were put together into one system rather than differentiating between two such apparently grossly different forms of responses [20]. Cannon was the first to describe the adrenal medullary responses to fear and anger and noted that the release of norepinephrine produced “strikingly bodily alteration, in which blood flow shifts away from the abdomen to the heart, lungs and limbs” [22]. Thus, Cannon's observations founded the physiologic basis (norepinephrine and sympathetic system) for fear and anger or for “fight or flight” responses. Later on, many studies have suggested that fear and anger are subsided by similar physiological arousal. Both fear and anger can induce sympathetic nervous system activation, and researchers have suggested that a pattern of physiological response characteristics of norepinephrine release is associated with fear and anger. For example, global increase in muscle tension, which indicates a general readiness for action or the level of effort currently being expended, is often regarded as a response for fear or anger, and this is also the original meaning of “arousal.” Toobey (1990) said that fear and anger can aid survival by influencing an organism to either flee for safety or fight to defend itself [39]. As such, we suggested that fear and anger might be two sides of the same coin [30]. Izard suggested that the individual will give a primary appraisal (comparison about his own resources with the environment) to decide flight or fight [22].

However, fear is a sensation about an object, such as a snake, and anger is due to a result of a behavior. Fear has been traditionally divided into several levels: automatic sense, physiological changes, attempts to escape, and subjective experience [28] (Figure 5). The automatic sensation level of fear, such as the fear of spiders, is frequently referred to as biological preparedness. Other uses of the word fear are actually new meanings developed from the biological level of fear [28]. In contrast, people are inclined to attribute the causes of their anger to controllable aspects of another person's behavior [37]. Thus, anger is developed later at the behavior level (Figure 5), which is due to appraisals about behaviors. Or anger is a reaction to the appraisal that an agent has done something blameworthy, which is the principal appraisal that underlies anger [4]. This might be the reason that object pictures cannot induce anger.

*Sadness might derive from disgust*. Sadness and disgust are distributed similarly on the valence and arousal dimensions (Figure 4(c)). However, disgust is a sensation felt towards an object, while sadness is at a conscious level of emotions, which arises from failure or loss with no hope of reinstating the goal [17], so sadness develops at the behavior level of “S-O-R” (Figure 5). *Sadness is similar to disgust in that they all have taken/eaten/experienced the disliked object/event*. However, sadness is a kind of conscious emotion which can only be experienced by humans or other high level animals, instead of lower level animals, such as insects. The lower level animals might not have the sad emotion. For example, people will be angry at somebody's mistreat for a baby, or people will be sad at the failure to get what they like. Thus, anger and sadness are not prototypical emotions, because they develop later and arise from higher level of cognitive process. However, anger is developed earlier than sadness, while anger is shared with all animal species, sadness might not be shared with lower level animals (e.g., insects).

*Surprise might also derive from fear*. Surprise is one of the most prevalent disagreement about basic emotions, and many people include it in their list of basic emotions, but surprise seems to have neither positive nor negative valence, so surprise is actually a cognitive state [4]. All objects have two features: whether it fits our needs (yes-like-joy; no-dislike-disgust) and whether it occurs as expected (surprise-fear) [9]. Surprise, as a kind of cognition, plays a major role in elicitation and intensification of emotions (Figure 5). For example, it is suggested that happiness equals unexpected joy (Happiness = Occurred–expected joy) [40]. So in the Western culture, surprise usually suggests unexpected happiness.

However, Jack et al. proposed that disgust and anger may be one emotion, and fear and surprise are one emotion [16]. If we look at the neurotransmitters, norapinephrine is the substrate for fear and anger (fight-or-flight) [35]. Disgust is due to serotonin in the digestive system, and sadness has also been linked to serotonin [32]. So anger might not have any relationship with disgust. At unconscious level, anger is due to cheating/harm, and disgust is due to decay; happiness is due to gain, and sadness is due to loss [41]. At the conscious level, Ekman said happiness is a goal that is attained, sadness is a failure to attain a goal, anger is an agent that causes a loss of a goal, and fear is an expectation of failure to achieve a goal [41]. In all, there might be five emotions: happy, fear, disgust, anger, and sad [42], which are due to conscious reappraisals about the results of behaviors. While prototypical emotions are due to unconscious perception about objects, other emotions, such as anger or sadness, are due to behaviors.

Even though emotional disorders are all at conscious level or subjective level, they might have problems in prototypical emotions. For example, major depressive disorders have major problems in the monoaminergic neuromodulators, and drug addictions have problems in dopaminergic problems. Just like what we proposed in our previous paper [3], almost all emotional disorders might be derived from the monoaminergic neuromodulators, and the first-line treatment for these diseases is still targeting monoaminergic neuromodulators. In addition, the levels of monoaminergic neuromodulators and event-related potentials can be used for the diagnosis for these diseases. So far, there are many reports about event-related potential changes in depressions and anxiety [43]; this paper might be the first one to probe into the changes from a basic emotional level.

## 4. Conclusion

Diagnosis of affective disorders is getting even harder now, and we have probed into the ways in the diagnosis previously [1, 3, 14, 25]. A better way to screen the affective disorder is using basic emotional theory [44, 45]. A widespread assumption in emotional theories is that there exist a limited number of basic emotions. Even though most psychologists agree upon the idea that there are some basic emotions, there is little agreement about how many emotions are basic, which emotions are basic, and why they are basic. In this paper, we used object pictures and ERPs to screen the basic emotions and emotional disorders and found that object pictures can induce only three basic emotions, joy, fear, and disgust. Anger and sadness emotions cannot be evoked by objects, and they can only be induced by someone's misbehavior. Therefore, we concluded that joy, fear, and disgust are three prototypical emotions, which can be combined to form many other emotions, like the three primary colors. We think this paper introduced a novel finding in the field of emotion, and this paper will bring a revolutionary impact on the field of emotional studies and bring interests from a broad readership.

In all, this study might be the first to suggest three prototypical basic emotions at the earliest developmental stage, which are joy, fear, and disgust. The prototypical emotions are evolved as the most basic emotions and form all other emotions like the three primary color. These emotions are automatic reactions and shared with all animal species. They are not consciously subjective emotions, which can only happen in human beings. Other emotions, such as anger and sadness, are developed later. Anger is still at the unconscious level and shared with animal species, while sadness might only happen in human being. So we concluded that only joy, fear, and disgust are evolutionarily the most prototypical emotions, which can form other emotions, like the three primary colors.

## 5. Materials and Methods

### 5.1. Participants

31 healthy (19 females, 12 males), right-handed college students from Sichuan Normal University with normal vision participated in this study. Participants' mean age was 21.2 ± 2.2 years (18-23 yrs). All subjects reported no history of neurological or psychiatric disorders. Written informed consent was obtained before the experiments, and the study was approved by the committee of ethnic board of Sichuan Normal University and the latest revision of the Declaration of Helsinki.

### 5.2. Stimuli

The stimulus material consisted of picture from the International Affective Picture System (IAPS) and the Chinese Affective Picture System (CAPS). The criteria for choosing pictures were that only objects were shown on the picture, and neither complicated scenery, human facial pictures, nor words were included. In order to avoid ambiguity of responses, pictures with only one featured object, such as a snake, cake, or fly, were preferred. 122 seventy pictures (72 from IAPS and 50 from CAPS) were pooled together. The pictures were presented in color, equated for luminance and contrast. IAPS stimuli included unpleasant, pleasant, and neutral objects. Pictures displaying facial or bodily expression or complex events and landscape are removed. To ensure that there was no luminance difference across the final images in the emotion pictures, we measured the luminance of each picture on the screen with a photometer. A randomized order and the subjects were asked to decide what basic emotions the picture can be induced, such as fear, anger, disgust, joy, surprise, and sad. Subjects were seated comfortably at about 75 cm from a 19 in screen in an electromagnetically shield room. The subjects were presented with a brief colored picture, which are randomized.

### 5.3. Design

Prior to the experiments, subjects were trained to be familiar with the experimental task through viewing 15 neutral pictures. Subjects were told to report what kind of emotions the pictures can induce “what kind of emotions can you feel about this picture”. The stimuli were presented on a 21 inch computer screen. Subjects were seated a 1 m distance from the screen with their head comfortably positioned in the chin and forehead. Participants were passively exposed the pictures and press the “empty space” key for “yes,” any other key for “neutral” to assess their subjective categorization and rating of the picture. Each picture was displayed on the screen for 500 ms, followed by 1 s rest interval with black screen. Pictures from each category of emotions were randomly presented. The participants first sorted out the pictures into the six emotion categories and one neutral category. Second, they rated the arousal and valence of their own emotional experience, as triggered by the displayed picture, on two independent 9-point Likert scales ranging from 1 (very unpleasant/not at all arousing) to 9 (very pleasant/very arousing).

### 5.4. EEG Data Acquisition

Brain electrical activity was recorded at 64 scalp sites using Ag/AgCl electrodes mounted on an elastic cap, with reference on FCz, and a ground electrode on the medial frontal aspect. The EEG were amplified using a 0.05 to 100 Hz bandpass and were continuously digitized at 1000 Hz/channel. All interelectrode impedances were maintained below 5 k*Ω*, and the data were referenced to the average of the left and right mastoids. Recordings were done in Brain Amp DC amplifiers (Brain Products, Germany).

### 5.5. Measurement and Analysis

The analysis of the neural mechanisms focused on ERP components elicited by the picture-induced emotions. The ERP was recorded 200 ms before the pictures were shown on the screen, and averaged epochs for the ERPs were 1,100 ms, including 200 ms prepicture array and 900 ms postpicture onset. Separate averages were computed for each subject at 5 neutral pictures. Contralateral waveform was calculated as the average of the left-sided electrodes to the right-sided items and of the right-sided electrodes to the left-side items. Ipsilateral waveforms were calculated as the average of the left-sided electrodes to the left-sided electrodes.

## Figures and Tables

**Figure 1:** Only three basic emotions can be activated by object pictures. (a) The distributions of responses from the object pictures from IAPS and CAPS show that joy, fear, and disgust are three major basic emotions. (b) Number of pictures for each categorized emotion. Pictures were categorized according to the emotion that gained more than half of the responses. (c) The average accuracy for each emotion is 67.3 ± 5.1% (*n* = 63) for neutral, 76.5 ± 3.9% (*n* = 32) for joy, 55.4 ± 3.7% (*n* = 16) for fear, and 71.4 ± 4.3% (*n* = 12) for disgust, respectively. (d) The averaged percentage of emotional responses (top label) for categorized neutral, joy, fear, and disgust pictures (left label).

**Figure 2:** The three prototypical emotions showed the fastest responses. (a) The procedure for the “Winner-takes-all” approach experiment. (b) The accuracy of the responses for each group of pictures. The side labels mean the group of pictures, and the top labels mean the responses for the 6 kinds of emotions. (c, d) The reaction times for joy, fear, and disgust are significantly shorter than those of the other three basic emotions (*p* < 0.01, one-way ANOVA). (e) The procedure for the “go/no-go protocol” experiment. The emotion picture was presented until the participant choose the space bar.

**Figure 3:** ERP studies of 6 basic emotions. (a) Typical ERP recordings at Pz. (b) Statistical analysis of averaged amplitudes of ERP recordings at P1, P2, and P3. (c) Relative amplitude ([relative peak = (categorized − neutral)/neutral) of ERP recordings at Pz. Statistical analysis showed that fear, joy, and disgust induced the earliest responses.

**Figure 4:** ERP studies of 6 basic emotions. (a) Topological distribution of ERP recordings at P1 shows that fear, joy, and disgust have the strongest P1 response at Pz points. (b) Valence and arousal distributions of the 6 categorized pictures showed that sadness and disgust overlapped, surprise and joy overlapped, and fear and anger overlapped. (c) Statistical analysis of valence and arousal showed that disgust and sadness have similar negative valence; fear and anger have similar arousal.

**Figure 5:** A schema shows that joy, fear, and disgust are three prototypical emotions. Emotions are developed at two major levels: unconscious and conscious. Like what Lazarus [14] said “I distinguish between two modes of appraisal: one automatic, unreflective, and unconscious; the other deliberate and conscious.” The lower level animals may not experience emotions consciously; they do have the prototypical emotions. The prototypical emotions are due to automatically sensation/perception about the objects, such as dizzy at height (fear), or nausea at a stool (disgust), or arousal at a sex nude body (joy). These three prototypical emotions fit for two primary needs: physiological need (valence: like–joy; dislike–disgust) and safety needs (arousal–fear) [19]. The unconscious appraisal can be divided into three levels: sensation-opinion-behaviors (S-O-R). Surprise is due to perception about the ways the object appears, while anger or sadness is due to behaviors that deals with the object.

## Data Availability

Original data are available if required.
